The article "Observation on cadavers and through ultrasonography using a 2 mm needle length for intradermal injections" was published in 2023. Journal: Skin Res Technol.

# Observation on cadavers and through ultrasonography using a 2 mm needle length for intradermal injections

**DOI:** 10.1111/srt.13529

**Published:** 2023-11-20

**Authors:** Kyu‐Ho Yi, Brian Lee, Michael James Kim, Seo‐Hyun Lee, Inneke Jane Hidajat, Ting Song Lim, Hyoung Moon Kim, Jin‐Hyun Kim

**Affiliations:** ^1^ Division in Anatomy and Developmental Biology Department of Oral Biology Human Identification Research Institute BK21 FOUR Project Yonsei University College of Dentistry 50–1 Yonsei‐ro, Seodaemun‐gu Seoul South Korea; ^2^ Maylin Clinic (Apgujeong) Seoul South Korea; ^3^ Department of Internal Medicine NewYork‐Presbyterian Brooklyn Methodist Hospital Brooklyn New York USA; ^4^ Aeon Medical and Aesthetic Centre Singapore Singapore; ^5^ Maylin Clinic (Yeouido) Seoul South Korea; ^6^ Department of Dermatology Faculty of Medicine Atma Jaya Catholic University of Indonesia Jakarta Indonesia; ^7^ Clique Clinic Kuala Lumpur Malaysia; ^8^ Maylin Clinic (Ilsan) Goyangsi South Korea

**Keywords:** Anatomy, intradermal injection, microneedle, polynucleotides, skin

## Abstract

**Background:**

An intradermal injection is a medical procedure that involves administering a small amount of medication or substance into the dermal layer of the skin. This research focused on identifying the most suitable injection needle for precise intradermal administration of skin boosters.

**Methods:**

The study involved conducting intradermal injections on four cadavers and participants using a 2 mm length, 34‐gauge needle (N‐Finders, Inc., South Korea). During the cadaveric study, the polynucleotide prefilled syringe was dyed green, and an anatomist performed dissections, removing only the skin layer. Ultrasonographic observations were carried out to ensure accurate intradermal injection placement.

**Results:**

In all four cadavers, the facial injections at the anterior cheek region were precisely administered intradermally at a 30‐degree injection angle. However, the 90‐degree injection was found just below the dermal layer upon skin layer removal.

**Discussion:**

The findings suggest that using a 2 mm needle length allows for easy and convenient intradermal injections.

## 1 INTRODUCTION

Although there is no precise consensus on the exact definition of skin boosters, their introduction is believed to have originated around 2015. Initially, skin boosters were developed using hyaluronic acid fillers with minimal crosslinking agents, specifically butanediol diglycidyl ether (BDDE), to enhance the skin's moisture levels. Since their inception, various skin booster products with diverse functions have been introduced to address and enhance different skin conditions.^1^ Due to the assertions made by many skin booster products, which include claims of skin regeneration, increased collagen production, improved elasticity, enhanced moisture, and whitening capabilities, the majority of these products are designed to target the dermal level of the skin.

The article "Observation on cadavers and through ultrasonography using a 2 mm needle length for intradermal injections" was published in 2023. Journal: Skin Res Technol.

An intradermal injection is a medical process involving the introduction of a small quantity of medication or substance into the dermal layer of the skin. The dermal layer, situated directly beneath the epidermis (the outermost skin layer), constitutes the second layer of the skin.^2^ This injection method is commonly employed for diagnostic applications, including conducting skin tests for allergies, tuberculosis, or specific vaccines that demand a distinctive administration approach. In the present day, numerous skin booster substances like hyaluronic acid, growth factors, Nevertheless, administering intradermal injections can present certain difficulties due to various reasons. The shallow depth of insertion, just below the skin's surface, requires precise needle placement into the dermal layer. Additionally, these injections can be more painful and uncomfortable compared to other types of injections because the dermal layer houses a higher density of nerve endings, leading to heightened sensitivity experienced by patients during the procedure. ^3^

Because of its close proximity to the epidermis, the dermal layer can frequently exhibit leakage through the hair follicles.^4^

The typical depth of facial skin varies anatomically, with the epidermis being relatively thin compared to other body parts, measuring approximately 0.1 to 0.5 mm in the facial area. On the other hand, the dermal layer in the facial region is thicker than the epidermis, ranging from 1 to 2 mm in depth. These measurements can also be influenced by ethnicity, as depicted in Figure 1, 5, 6.

**FIGURE 1:** The variation in skin thickness between Asians (A) and Caucasians (B). The Asian population generally exhibits approximately 0.1 mm greater skin thickness than Caucasians. The skin thickness range differs, varying from 1 to 2 mm in depth, depending on ethnicity.

Based on mathematical analysis, it is feasible to achieve a consistent injection depth of 1 mm into the dermal layer using a 2 mm needle length with a full needle injection angle of 30 degrees.

The research investigated the most suitable injection needle for skin‐booster injections to ensure precise intradermal administration.

## 2 MATERIAL AND METHOD

We performed cadaveric injections using a 2 mm length, 34‐gauge needle (N‐Finders, Inc., South Korea) on four cadavers. During the cadaveric study, the polynucleotide (PN) prefilled syringe was colored green, and an anatomist conducted the dissection, removing only the skin layer.

The article "Observation on cadavers and through ultrasonography using a 2 mm needle length for intradermal injections" was published in 2023. Journal: Skin Res Technol.

Additionally, we observed four participants with ultrasonography during intradermal injections of PN. The patients received a series of 1cc PN injections (Rejuran‐s; Pharmareasearch Products, Inc., Seongnam, Republic of Korea) with a concentration of 20 mg/mL. Using a 34‐gauge 2 mm needle and administering the intradermal injection at a 30‐degree angle, approximately 0.02–0.03cc of PN was injected (Figure 2).

**FIGURE 2:** The administration of polynucleotide through a 34‐gauge 2 mm needle at a 30‐degree angle, resulting in an injection of approximately 0.02–0.03 cc at each point.

The exact location of the dermal injection was observed through ultrasonography images, which were obtained using a real‐time two‐dimensional B‐mode US device equipped with a high‐frequency (18 MHz) linear transducer (Sonimage HS1, KONICA MINOLTA, Tokyo, Japan).

## 3 RESULT

In all four cadavers, the facial injections at the anterior cheek region were accurately located intradermally with a 30‐degree injection angle. Conversely, the 90‐degree injection was situated just below the dermal layer, as observed after removing the skin layer (Figure 3).

**FIGURE 3:** The anterior cheek of the cadaver was injected with green dye and dissected with the removal of the dermal layer. Polynucleotide injections were carried out at 90 degrees (A) and 30 degrees (B) using a 2 mm needle length (N‐Finders, Inc., South Korea). Intradermal injections were observed inside the dermal level when the skin was removed, while subdermal injections were observed with the 90‐degree injection.

Ultrasonographic observation revealed that all intradermal injections appeared to be properly placed within the dermal layer when administered at a 30‐degree angle using a 2 mm, 34‐gauge needle at the anterior cheek region (Figure 4).

**FIGURE 4:** The figure depicts ultrasonography results, where posterior shadowing (A, circled) is observed. The polynucleotide was injected at a distance of 1 cm (B, white arrows).

## 4 DISCUSSION

Starting from 2015, the skincare and cosmetic surgery market began using the term “skin booster” when introducing products like “Restylane Vital” and “Restylane Vital Light,” which are hyaluronic acid fillers aimed at supplying HA to the dermal layer for skin rejuvenation and wrinkle reduction.^5^ Prior to this, HA fillers were primarily utilized for increasing volume, but the concept of using HA fillers as skin boosters emerged with the objective of enhancing the skin condition by improving the dermal layer's extracellular matrix.

Numerous research studies are currently investigating skin boosters to comprehend their mechanisms and effectiveness. These studies encompass a wide range of substances, including hyaluronic acid fillers, botulinum toxin, poly‐L‐lactic acid (PLLA), poly‐D‐lactic acid (PDLA), poly‐dioxanone (PDO), polynucleotide (PN), polydeoxynucleotides (PDRN), growth factors, exosomes, and various amino acids.^5^, ^6^, ^7^ Several subsequent studies have demonstrated that intradermal injections yield skin‐lifting effects, pore reduction, enhanced skin tension, and reductions in acne, sebum secretion, and sweating through eccrine glands.^8^

The article "Observation on cadavers and through ultrasonography using a 2 mm needle length for intradermal injections" was published in 2023. Journal: Skin Res Technol.

Yet, intradermal injections pose certain challenges due to shallow depth requirements. The needle must be precisely inserted into the dermal layer, situated just beneath the skin's surface.^9^ Moreover, intradermal injections often induce more pain and discomfort than other types of injections because the dermal layer houses a higher density of nerve endings compared to subcutaneous tissue or muscle, leading to increased patient sensitivity during the procedure. Some studies have suggested that blocking the secretion of calcitonin gene‐related peptide and vasoactive interstitial peptides can reduce flushing, promote collagen synthesis, and enhance skin texture. However, intradermal injection may elicit complaints of pain akin to a feeling of being “torn up.” One potential drawback of intradermal injection in comparison to intramuscular injection is the likelihood of heightened pain, as the dermal layer is in close proximity to the epidermis and may occasionally seep out from hair follicles.^10^

In accordance with Poiseuille's law, the flow rate is inversely proportional to the length of the tubing of the needle. In simpler terms, when the needle is shorter, the flow rate is faster under constant pressure. Additionally, fluid viscosity is also inversely proportional to the flow rate, indicating that lower fluid viscosity results in a faster flow rate (Figure 5).

**FIGURE 5:** As per Poiseuille's law, the flow rate is inversely proportional to the length of the needle tubing and fluid viscosity.

Injectable skin boosters often consist of biostimulators like polymers, such as polynucleotide and polyribonucleotide, along with non‐crosslinked or minimally crosslinked hyaluronic acid, which are commonly used for injection as skin boosters. In the context of skin booster injections, the frequently employed microneedle has a size of 33‐gauge and a length of 4 mm, suitable for subdermal layer injections, and can be adjusted for intradermal injections by modifying the injection angle, while a 2 mm needle is primarily intended for intradermal use (Figure 6).

**FIGURE 6:** In the realm of skin booster injections, a commonly used 33‐gauge, 4 mm microneedle (A) is versatile for subdermal and intradermal injections with adjustments to the injection angle, while a 2 mm needle (N‐Finders, Inc., South Korea) is primarily designed for intradermal use (B).

The article "Observation on cadavers and through ultrasonography using a 2 mm needle length for intradermal injections" was published in 2023. Journal: Skin Res Technol.

The typical depth of facial skin varies anatomically. The epidermis and dermis in the facial area is comparatively thinner than in other body parts, measuring approximately 0.1 to 0.5 mm. In contrast, the dermis in the facial region is thicker than the epidermis, ranging from 1 to 2 mm in depth, and this can vary depending on a person's ethnicity.^11^, ^12^

The study has revealed the ease and convenience of performing intradermal injections using a 2 mm needle length.

## CONFLICT OF INTEREST STATEMENT

The authors have all considered the conflict of interest statement included in “Author Guidelines”. To the best of our knowledge, no aspect of the authors’ current personal or professional life might significantly affect the views presented on this manuscript. The authors declare no conflicts of interest.

## Data Availability

The data that support the findings of this study are available from the corresponding author upon reasonable request.
